# An Ideal Approach for Enhancing 5-Fluorouracil Anticancer Efficacy by Nanoemulsion for Cytotoxicity against a Human Hepatoma Cell Line (HepG2 Cells)

This article has been retracted.

**DOI:** 10.1155/2022/4094132

**Published:** 2022-06-17

**Authors:** Jamal Moideen Muthu Mohamed, Fazil Ahamad, Mohamed El-Sherbiny, Hasnaa Ali Ebrahim, Mohamed Ahmed Eladl, Amal F. Dawood, S. T. Sheik Abdul Khader, Karuppaiyan Kavitha, Dawit Mamiru Teressa

**Affiliations:** ^1^College of Pharmacy, Shri Indra Ganesan Institute of Medical Science, Manikandam, Tiruchirapalli, 620012 Tamil Nadu, India; ^2^Department of Anesthesia Technology, College of Applied Medical Sciences in Jubail, Imam Abdulrahman Bin Faisal University, P.O. Box 4030, Jubail, Saudi Arabia; ^3^Department of Basic Medical Sciences, College of Medicine, AlMaarefa University, P.O. Box 71666, Riyadh 11597, Saudi Arabia; ^4^Department of Basic Medical Sciences, College of Medicine, Princess Nourah bint Abdulrahman University, P.O. Box 84428, Riyadh 11671, Saudi Arabia; ^5^Department of Basic Medical Sciences, College of Medicine, University of Sharjah, Sharjah, UAE; ^6^Department of Pharmaceutical Technology, BIT Campus, Anna University, Tiruchirappalli, 620024 Tamil Nadu, India; ^7^Department of Chemical Engineering, College of Biological and Chemical Engineering, Addis Ababa Science and Technology University, Addis Ababa, Ethiopia

## Abstract

The core objectives of the research were to prepare 5-fluorouracil nanoemulsion (FU-NE) and to evaluate the physiochemical properties and to study the i*n vitro* antiproliferation in HepG2 cell lines. The physiochemical parameters determined were compatibility, particle size (PS), polydispersity index (PDI), zeta potential (ZP), density, surface tension (ST), pH, viscosity, *in vitro* release of FU, cytotoxicity, and apoptosis study. The prepared FU-NE3 was stable, sterile, and homogeneous. On the HepG2 (120 *μ*g.mL^−1^) cells, *in vitro* cytotoxicity was obtained at IC_50_ concentration. Apoptosis examination by AO/EBand Hoechst staining shows that the majority of cell demise was caused by apoptosis, with a tiny fraction of necrosis. Hence, this investigation concluded that the developed FU-NE has now desirable characteristics for drug delivery to the cancer cell and may be screened for the *in vivo* colorectal anticancer activity.

## 1. Introduction

Colon targeting drug delivery has several advantages in treating the colon diseases such as ulcerative colitis and colorectal cancer that are more effective area. This type of drug delivery is very essential by preventing and destroying of drug from stomach acid and from metabolism by pancreatic enzyme which slightly affected the colon [1].

Colorectal cancer (CRC) exists a tumour that progress at the colon or rectum. Depending on the organ involved, it is also called as colon rectal cancer. CRC recorded as the third and second causing cancer in males and females, respectively, with the third highest fatality rate of all cancers worldwide. The durable ulcerative colitis, colon cysts, and hereditary origins contribute to CRC, and it is most commonly diagnosed in people between the ages of 60 and 80. Polyps in the colon are also responsible for cancer cell proliferation, and there are three types of polyps: adenomatous (precancerous), inflammatory polyps, and hyperplastic polyps (cancerous condition). CRC is caused by polyps greater than one centimeter in diameter or the presence of two or more polyps [2, 3]. Adenomatous polyp cell dysplasia is a kind of adenomatous polyp cell that is not malignant yet causes CRC. Polyps that have spread to the blood or lymph arteries, lymph nodes, or other organs are cancerous polyps. 5-Fluorouracil (FU) is a pyrimidine analogue that is used in the treatment of cancer. It is a suicide inhibitor that operates by inhibiting thymidylate synthase in an irreversible manner. It is one of a class of medications known as antimetabolites. As a pyrimidine analogue, it is converted inside the cell into a variety of cytotoxic metabolites, which are subsequently integrated into DNA and RNA, causing cell cycle arrest and death by limiting the cell's capacity to generate DNA. It is an S-phase drug that only works during specified cell cycles [4]. The drug has been demonstrated to suppress the function of the exosome complex, an endonuclease complex whose activity is required for cell viability, in addition to being integrated DNA and RNA.

Drugs that are weakly acidic or basic and insufficiently water soluble have low solubility and bioavailability, according to the pharmaceutical industry. Micronization, nanosizing, amorphous to crystalline form conversion, wettability improvement, liposomal delivery [5], and formation of salts and prodrugs are just a few of the physicochemical processes that might help with solubility.

A nanoemulsion (NE) is a liquid dispersion that has an oil phase and a water phase, as well as a thermodynamically or kinetically stable surfactant [6]. The dispersed phase, which has very low oil/water interfacial tension, is made up of small particles or droplets with a size of 5-200 nm. NEs are transparent because 25% is the average droplet size of the wavelength that could be visible light [7].

Nanoemulsions, unlike microemulsions, may be generated with a lower surfactant content (usually 3–10 percent). Because nanoemulsions have a greater in free energy and surface area, they are a more efficient means of transport. Foams, creams, liquids, and sprays are just a few of the options [8]. They are safe to use on the skin and mucous membranes because they are nontoxic and nonirritating. If the formulation contains biocompatible surfactants, it can be taken orally.

Nanomedicine has emerged as a new branch of medicine in the recent decade, with the potential to solve some of the problems linked with existing chemotherapy treatment such as severe chemotherapeutic drug resistance and drug side effects. For reducing systemic toxicity induced by chemotherapy treatments, several nanocontainers and drug delivery mechanisms have been proposed [9]. Liposomes, polymeric micelles, hollow particles, emulsion droplets, and other forms are commonly utilised to encapsulate drugs. The encapsulation method has the ability to significantly increase drug concentration in an aqueous environment and breathe new life into bioactive molecules that had previously been written off due to their least soluble in aqueous environment.

## 2. Materials and Methods

### 2.1. Materials, Regents, and Cell Lines

The following chemicals was purchased: 5-fluorouracil (FU), Eudragit® RS PO (EuDR; 98.9% of purity; SpectroChem Pvt. Ltd., Maharashtra, India), PEG, castor oil, and Tween 80 (S.D. Fine Chem. Pvt. Ltd., Mumbai, India). The cell line HepG2 (human hepatoma cell line) was purchased from National Animal Cell repository at National Centre for Cell Science (NCCS), Pune. Then, the cells were grown in T25 flasks as a monolayer in the presence of DMEM, i.e., Dulbecco's Modified Eagle Medium (Sigma-Aldrich, USA) accompanied with fetal bovine serum (10%), 50 *μ*g/mL of antibiotic and maintained at 5% humidified CO_2_ incubator (Thermo Scientific, USA) in 37°C of temperature. Analytics grades of chemicals and reagents were used for this investigation.

### 2.2. Compatibility Study

The Fourier transform infrared (FTIR) spectrometer was utilised to conduct compatibility of Eudragit® RS PO, surfactants, and preparation. Briefly, the samples were combined with potassium bromide (KBr; 1 : 10) and squeezed in a hydraulic press under 10 tons of pressure to generate translucent KBr pellets, which were subsequently scanned by FTIR in 4000 to 400 cm^−1^ wave number range. In the same way, the dried formulation was investigated [10].

### 2.3. Preparation of FU-Nanoemulsion (FU-NE)

The FU-loaded nanoemulsion was prepared as shown in Table 1 by dispersing 5-FU and 50 mg of EuDR (1 : 1) in methanol (20 mL) using a bath sonicator, then adding 80 *μ*L of castor oil to the methanolic FU solution. The aqueous phase was made by mixing Tween 80 (0.1 mL) and PEG 400 (0.1 mL) in double distilled water [11]. Addition of aqueous phase to the oil phase and stirred magnetically (REMI2) at 500 RPM for 10 min followed by sonication (Sonics & Materials VCX 750, Inc., Newtown, USA) at 20 kHz for 5 min (pulse rate of 5/1 sec and amplitude 35%). The stable microemulsion was homogenized for 5 minutes at 14,500 rpm in an Ultra Turrax T25 homogenizer (IKA, Ohio, USA). The resultant nanoemulsion (FU-NE) and the resultant solution were cooled down to 4°C to obtain FU-NE.

### 2.4. Characterization of FU-NE

#### 2.4.1. Drug Content (DC) and Entrapment Efficiency (% EE)

After being disrupted with methanol, the amount of FU encapsulated in the dialyzed FU-NE was measured. An aliquot of FU-NE was combined with an adequate amount of methanol and then covered with a parafilm to prevent methanol evaporation to form a clear solution [12]. After appropriate dilution, the concentration of FU was determined spectrophotometrically at 266 nm (Model No. UV 2401 (PC), S.220V, Shimadzu Corporation, Japan). There was no interference from blank NE at this frequency. The EE was estimated using the formula below.

(1) $$\begin{array}{c} \%\text{EE}=\frac{\left(\text{Actual DC in FU}‐\text{NE}\right)}{\left(\text{Theoretical DC in FU}‐\text{NE}\right)}\times 100. \end{array}$$

#### 2.4.2. Dynamic Light Scattering

The particle size (PS; nm), zeta potential (ZP), and polydispersity index (PDI) of FU-NE preparation were assessed by photon correlation spectroscopy by Zetasizer Ver. 6.20 (Malvern Instruments) and were utilised to evaluate the droplet size of the samples [13]. To eliminate multiscattering effects and experimental slips, diluted with distilled water, the formulation was filtered using a 0.22 membrane filter. At a temperature of 25°C, light scattering was measured at a scattering angle of 90^o^. PDI is a dimensionless measure of a particle size distribution's broadness that may be used to assess nano-sized preparations [14].

#### 2.4.3. Dispersibility, Density, Viscosity, pH, and Surface Tension (ST) of FU-NE

The efficiency of oral FU-NE was determined using a dissolution apparatus. At 37 ± 0.5°C, addition of one mL of each formulation to 500 mL of distilled water. Gentle agitation was achieved using a typical stainless steel dissolving paddle moving at 50 rpm [15]. The compositions in vitro performance were assessed visually.

The method explained by Nejadmansouri et al. was used to determine the density of nanoemulsion. Briefly, the FU-NE was filled to the specified level (10 mL) using pycnometer, and the weight was calculated [16]. It was done in the same way with water and weighed. The density of FU-NE and water was compared, and the density of FU-NE was calculated.

The ST of FU-NE was assessed using the drop count method using stalagmometer (Borosil). The provided liquid was drawn into the drop pipette up to a mark in this approach [16]. The number of droplets created as the liquid level lowers is counted by holding the pipette vertically. The following formula was used to compute the relative surface tension of the samples.

(2) $$\begin{array}{c} \text{ST}=\frac{\rho \text{FU}‐\text{NE}\times \;\eta \text{w}}{\rho \text{w}\times \eta \text{PU}‐\text{NE}}, \end{array}$$

where *ρ*FU-NE is the density of FU-NE, *η*w is the viscosity of distilled water, *ρ*w is the density of water, and *η*PU-NE is the viscosity of FU-NE.

As specified in our previous study, the viscosity of the produced FU-NE was evaluated using a Model No. CSAP2000 + L Brookfield viscometer (Brookfield Engineering Lab., USA) at 37 ± 0.5°C with 50 rpm using spindle no. 1 [17]. A calibrated pH meter was used to measure the apparent pH of the formulations in triplicate at 25°C, and the pH was determined by dipping a glass electrode into the FU-NE.

#### 2.4.4. Morphology of FU-NE

A TECHNAI 10 transmission electron microscope (TEM) is an efficient to produce better resolution, and operating at 200 kV was used to analyze the morphology and surface structure of the FU-NE [18] (Technai 10, Philips). A drop of NE was placed to the film grid and inspected after it dried to make the TEM observations.

#### 2.4.5. *In Vitro* FU Release Study

The *in vitro* drug dissolution research of the FU-NE formulation was carried out using a dialysis membrane (Himedia®, India; avg. flat width of 25.27 mm; avg. dm of 15.9 mm) that had been soaked for 12 hours with pH 7.4 phosphate buffer. The volume of FU-NE preparation corresponding to 5 mg FU had distributed in 5 mL of phosphate buffer and put in an activated membrane bag with both ends sealed. The dialysis bag was then placed in the PBS containing beaker and set up in the magnetic stirrer (REMI 2) (DA-3, Veego Scientific Devices, Mumbai, India), with the magnetic bead being inserted in the jar holding 100 mL dissolving media. The temperature in the experiment was maintained at 37 ± 0.5°C with 100 rpm stirring. To maintain the sink state, 1 mL aliquots were taken at predetermined intervals and replenished with an equivalent volume of fresh buffer [19]. UV-Spectrophotometry (S.220V, UV-2401(PC), Shimadzu Corporation, Japan) was used to examine all samples at 266 nm. To evaluate the drug release properties of FU-NE formulations, the experiment was repeated three times. The release of the drug was compared to pure FU, which was suspended in 5 mL of buffer and studied in the same way as FU-NE. The varied release mechanisms of controlled drug delivery systems were expected to be reflected in drug release kinetics. As a result, five kinetics models were used to assess the *in vitro* statistics in order to choose the top ideal equation based on our past research.

### 2.5. In Vitro Cytotoxicity Assay

The *in vitro* cytotoxicity experiments are important for determining intrinsic cytotoxicity, inhibitory concentration ranges, genotoxicity, and programmed cell death, among other related cell death. It could compare the response of a single chemical in several systems or numerous compounds in a single system by determining the IC_50_ value (half maximum inhibitory concentration).

#### 2.5.1. Plating Out of Cells for *In Vitro* Assay

The trypsinized HepG2 cells were collected from the T25 flask, and the cell suspension was centrifuged to yield a pellet. The cells were then resuspended in growth media and calculated by a hemocytometer, and the counting zone was covered by the cover slip. Between the counting chamber and the cover slip, the resuspended cell suspension was introduced [20]. The cells present in the four sides of the WBC counter were counted, and the average number of cells was computed using a light microscope. From the average number of cells, the volume of cell suspension to be added in the 96 well plate to get 5000 cells was calculated.

(3) $$\begin{array}{c} \text{Average number of cells}=\frac{\left(\text{cells in A}+\text{cells in B}+\text{cells in C}+\text{cells in D}\right)}{4},\\ \text{Volume of cell suspension to get }5000\text{ cells}=\text{Avg}.\text{no of cells}\times \text{Total Volume}\times \text{Dilution Factor}\times \text{Conversion factor}. \end{array}$$

All of the wells received 100 *μ*L of growth medium. After the cells have been counted, a cell suspension containing 5000 cells is added to each well of a 96-well plate, with the exception of the first column, which is left blank. The plate was incubate using CO_2_ incubator for 24 hours at 37°C in a humidified CO_2_ environment of 5% [21].

#### 2.5.2. MTT Addition

The MTT (3-(4,5-dimethylthiazol-2-yl)-2,5-diphenyltetrazolium bromide) study was conducted on HepG2 cells. The cells were cultivated at a mass of 5 × 10^3^ cells in 96-well plates. The DMSO solvent was used as a control, using cells.mL^−1^ in 200 L.well^−1^. Prepared FU-NEs were treated with 20 mL.well^−1^ MTT reagent (20 mL.well^−1^) and incubated for further 4 hours at 37°C after a 24 h incubation period. The purple formazan product was diluted in all of the wells by adding 100 mL of DMSO solvent [22]. Using a plate reader, the aforementioned solution absorption was measured at 570 nm using a 630 nm reference filter (iMark, Bio-Rad, USA). This data was used to compute the % inhibition, which was derived by the following formula.

(4) $$\begin{array}{c} \text{Inhibition }\left(\%\right)=\frac{\left(\text{Control OD}-\text{Sample OD}\right)}{\text{Control OD}}\times 100. \end{array}$$

The IC_50_ concentration which will be calculated from the MTT assay would be necessary to kill 50% of the cells.

*(1) Acridine Orange/Ethidium Bromide (AO/EB) Stain*. The 5 × 10^4^ HepG2 cells were planted into 6-well culture plates and allowed to develop to 80% union. The cells were subsequently cultivated for 24 h with the IC_50_ concentration (derived from the MTT assay) of FU-NE (which yielded the greatest results in the MTT assay). Phosphate buffered saline (PBS) was used to suspend the cells after trypsinization. Before being covered with a cover slip, a drip of cell dispersion was put onto a glass slide and treated with AO/EB (Sigma Chemical Co., St. Louis, USA). The dyed cells were then viewed at 400x magnification with a Carl Zeiss fluorescent microscope (Jena, Germany) equipped with a filter range of 377–355 nm [13]. The number of cells with pathogenic alterations was determined.

*(2) Hoechst Stain*. Following trypsinization, the cell dispersion was treated with Hoechst 33258 stain and incubated for 15 minutes at 37°C, as reported by Moideen et al. [14]. The cells were formerly examined under a fluorescent microscope at a magnification of 400x to assess the percentage of cells with pathogenic changes.

*(3) Stability Study*. The physicochemical stability of an optimal formulation of FU-NE (F3) in a stability compartment (Wadegati TM Labe Quip (P) Ltd., Model No. HTC-3003, Andheri (E), Mumbai, India) for 3 months at 45 ± 0.5°C and 60 ± 5% RH. FU-NE examined physical changes, DC, PS, ZP, and *in vitro* drug release at 1-month intervals [13].

## 3. Results and Discussion

### 3.1. FT-IR Outcomes

The FTIR spectrum of the FU, polymers show in Figure 1, where FU make known the numeral of typical bands signifying O-H stretching (alcohol, 3403.93 and 2924.56 cm^−1^), C=O stretching (1737.54 cm^−1^), C-H bending (1446.31, 1365.22, 888.38, and 721.33 cm^−1^), and stretching vibration [23].

The characteristic bands of all, castor oil, Tween 80, PEG 400, and Eudra RS PO, demonstrate that O-H extending vibration (3403.93, 3481.50, 3308.23, and 3437.46 cm^−1^) relating to the samples vanished and C=O stretching (1737.54 cm^−1^) extending vibration (1641.54, 1644.65, 1631.43, and 1638.95 cm^−1^) attributable to FU found that decreases wavelength with FU-NE proposed the development of the complex by hydrogen bonding shown in Figures 1(b)–1(f). The solo peak detected at 2360.82 and 2078.03 cm^−1^ (C-H prolonging) might represent the FU excipient complexing option site. Similarly, the nonappearance of the N-H extending band at 3442 cm^−1^ is demonstrated by FU-NE, implying hydrogen bonding (intermolecular) among the FU and the polymer. The outcome of this study promising is that there is no interaction with the excipients that had been compatible with the FU and the prepared FU-NE.

### 3.2. DC and % EE

The FU-NE had a DC of 95.36 ± 0.31 to 98.43 ± 0.32 mg.mL^−1^ and a percent EE of 91.22 ± 0.46 and 94.46 ± 0.51 percent, respectively (Table 2). The high percent EE values are due to the lipophilicity of FU, which permits it to be well absorbed into lipid bilayers in all FU-NE preparations [24]. The DC of FU-NEs in chosen batch F3 was 98.26 ± 0.35 mg.mL^−1^ of FU-NEs, and the percent EE of chosen batch F3 was 91.07 ± 0.61%. It was detected that the particular batch F3 exhibited the highest DC with ideal % EE due to improve in native character of drug and polymer with oil ratio (1 : 1 : 0.06).

### 3.3. DLS Outcome

Table 2 displays the average PS, PDI, and ZP values of FU-NE ranged from 125.76 ± 1.62 to 197.23 ± 2.87 nm with the PDI of 0.278 ± 0.076 to 0.137 ± 0.054. This indicates that prepared FU-NEs were of mono dispersion and only available in a limited number of locations (Figures 2(a) and 2(b)). The ZP value of F3 had a −20.9 ± 0.76, indicating that the formulation was stable throughout the period.

### 3.4. Physical Properties

The dispersibility test was carried out in a dissolving equipment, and the results revealed a clear transparent nanoemulsion formulation (Figure 2(c)). The density of all formulations was measured with a pycnometer, and the findings are listed in Table 3. The formulation's density is determined to be between 0.788 g/cm^3^ and 0.997 g/cm^3^. The density of NE3 was determined to be 0.7881 g/m^3^. A stalagmometer was used to determine the surface tension of all formulations, and the results were tabulated [24]. The formulations' surface tension was determined to be between 0.4387 and 0.4472 dynes/cm. Table 3 shows the results of calculating the pH of all formulations using a calibrated pH meter. The pH of the formulations ranged from 6.92 to 7.1. The pH of NE 3 was found to be 7.1.

Due to the existence of vesicular spherical structures with a large hydrodynamic volume, the FU-NE dispersions had a higher viscosity value than water [25]. F3 FU-NEs had a viscosity of 1.12 cP, which was much lower than that of FU-NEs (2.054 ± 0.65 cP). However, when shear rates rise, the viscosity rises as well, showing shear thickening behaviour. The viscosity was Newtonian because electrostatic repulsion impeded the formation of the interparticle structure at low shear rates. The shear rate was higher than 120 s1 according to Bai and Rai; however, the attraction of NE dispersions increased, causing the viscosity to consistently increase (2021). Furthermore, when the shear rate increases, the viscosity of NE dispersions increases abruptly, which might be owing to increased particle contact caused by the fast rotation speed [11].

### 3.5. TEM

As shown in Figure 2(d), a TEM analysis was performed on a chosen batch (F3) of FU-NEs with a drug-to-polymer proportion of 1 : 1. In the TEM of the FU-NEs, the boundary and centre of well-established globular smooth outer surface structures with spherical form can be seen. A lighter core was exposed, surrounded by a denser boundary that exactly ringed the centre. When a thin polymer coating was hydrated, it forms an encircled vesicular complex that allows the system to succeed with stabile by depressing over-all free energy [26].

### 3.6. *In Vitro* Drug Release

Each batch's FU release was accomplished by inserting a dialysis membrane into a dissolving instrument and soaking it in phosphate buffer for 12 hours (pH 7.4). As indicated in Figure 3(a), the cumulative FU release of all batches ranged from 72.72 ± 3.32 to 87.23 ± 3.12%. For 12 hours, the drug release of a chosen batch FU-NE3 and pure FU was determined to 87.23 ± 3.12 and 12.31 ± 0.31%, respectively. The FU-NEs have the ability to deliver the medicine in a regulated manner, as demonstrated in this study. As a result of the improved solubility of FU, continuous/uninterrupted drug release over a lengthy period of time may be obtained [27].

Table 4 shows that for improved batch FU-NEs, the Higuchi equation with the maximum linearity (*R*^2^ = 0.9926) best characterized *in vitro* drug release. The drug released together erosion and diffusion (non-Fickian diffusion) is indicated by the slope of the Korsmeyer-Peppas equation being more than 0.5 but less than 0.85 [28].

### 3.7. Culture of HepG2 Cell Line

#### 3.7.1. *In Vitro* Cytotoxicity Assay

In a T25 culture flask, a monolayer of HepG2 cancer cells was grown to 80% confluency. The inverted microscope was used to view live cells clinging to the bottom of the flask, as illustrated in Figure 3(b). The effects of a nanoemulsion of FU on a HepG2 cell line cultivated in a 96-well plate were investigated. The cells were treated with FU-NE3 for 24 hours at different doses ranging from 0 to 200 *μ*g/mL. The MTT assay revealed that FU-NE3 inhibited the development of HepG2 cell lines in a dose-dependent manner [29]. Only 120 *μ*g/mL FU-NE concentration was required after 24-hour treatment to kill half of the cells and achieve half maximum inhibitory concentration (IC_50_).

### 3.8. Mechanism of HepG2 Cell Death

#### 3.8.1. Outcome from AO/EB Stain

AO/EB dual stains were exhibited to confirm the apoptotic morphologies induced by FU-NEs [30]. According to the morphological properties of nuclei, three types of cytological alterations were discovered. Late apoptotic cells (Figure 4(a)) showed orange to red fluorescing nuclei and compressed or broken chromatin; necrotic cells were minimal chromatin fragmentation or condensation, were swollen, and had orange to red fluorescing nuclei. The second late apoptotic cell deaths were primarily found among them, as illustrated in Figure 4(c). The morphological alterations seen by this staining approach after 24 hours of treatment with FU-NE3 show that the cells were committed to death by both apoptosis and necrosis. However, in comparison to necrosis, a large percentage of cells perished by the apoptotic method of cell death, as illustrated in Figures 4(a) and 4(d).

### 3.9. Outcome from Hoechst Staining

DNA breakage, chromatin condensation and marginalisation, membrane blebbing, cell shrinkage, and cell fragmentation into membrane-enclosed vesicles or apoptotic bodies, which are phagocytosed by macrophages, are all signs of apoptosis [31]. The determination of apoptosis at a fundamental level, Hoechst staining has been recommended. The cells were evaluated for gross cytological alterations after being treated with FU-NE3 at the IC_50_ concentration for 24 hours. The treated cells shown (Figure 4(b)) the abovementioned microscopic cytological alterations associated with apoptosis, as well as late apoptosis-related dot-like chromatin. A few cells, however, showed signs of necrotic death.  Figure 4(e) depicts the quantities of normal and diseased cells calculated in the control and FU-NE3 treated groups.

### 3.10. Stability of FU-NE

The FU-NE was preserved for additional characterization and stability testing.  Table 5 shows that at ±0.5°C and 60% RH, FU-NE3 remained constant for 6 months. Merely a little increase in PS and PDI was detected after storage (161.11 ± 4.92 nm and 0.215 ± 0.086, respectively). After storage, the DC, percent EE, ZP, and in vitro drug release of FU were virtually identical to those before storage, with values of 98.43 ± 0.32 and 89.33 ± 1.95, 91.22 ± 0.46 and 83.67 ± 2.76, 20.90 ± 0.76 mV and −15.35 ± 1.36 mV, and 87.23 ± 3.12 and 95.33 ± 5.66%, respectively. This implies that when held at 4°C, FU-NE3 has a good physical stability [32].

## 4. Conclusion

The prepared 5-fluorouracil nanoemulsions may be used to treat colorectal cancer. The drug and excipients' compatibility was investigated. The methanol content was varied to create the formulations. FTIR, PS analysis, ZP, and TEM were used to characterize the formulations. *In vitro* drug release by dissolving research was used to determine drug release. Biocompatible particles are those with a diameter of less than 200 nm and a particle size of less than 126 nm. On the concentration of 120 g/ml, the *in vitro* cytotoxicity test was used to assess the suppression of cell growth for various concentrations and the IC_50_. AO/EB and Hoechst staining procedures were used to examine the morphology of cell death. As an outcome, cell death by apoptosis was discovered in the tested cells. It was tested and shown to have less necrosis and to be particularly efficient in killing cancer cells. As a result, we believe that the produced 5-fluorouracil nanoemulsion has demonstrated desirable *in vitro* features for drug delivery to cancer cells and might be tested *in vivo* for colorectal cancer targeting.

## Figures and Tables

**Figure 1:** The FTIR spectrum of (a) pure FU, (b) castor oil, (c) PEG 400, (d) Eudragit® RS PO, (e) physical mixture, and (f) FU-NE.

**Figure 2:** DLS result of (a) Avg. PS, (b) ZP, (c) dispersibility, and (d) TEM image of FU-NE3.

**Figure 3:** *In vitro* FU release from (a) pure FU and FU-NEs, and (b) *in vitro* cytotoxicity graph of FU-NE3 against HepG2 cell line (mean ± SD, *n* = 3).

**Figure 4:** (a) AO/EB and (b) Hoechst staining of HepG2 cells; (c) various morphological changes observed from AO/EB staining; (d) percent of alive, apoptotic, and necrotic cells of HepG2 cells subsequent 24 h exposed with HepG2 cells. (d) AO/EB and (e) Hoechst stain observed in fluorescent microscope of control and pure FU; ^∗∗∗^*p* < 0.001 and ^∗∗^*p* < 0.05 reflect major variances related with control, and both are tested using the student *t*-test.

**Table 1:** Composition of FU-NEs.

S. no	Components	FU-NE		
		F1	F2	F3
1	FU (mg)	50	50	50
2	EuDR (mg)	100	75	50
3	Methanol (mL)	20	5	5
4	Castor oil (*μ*L)	80	80	80
7	Tween80 (mL)	0.1	0.1	0.1
6	PEG 400 (mL)	0.1	0.1	0.1
7	Double distilled water (mL)	60	60	60

**Table 2:** Composition and characterization of ITZ-nPEV batches.

Preparations	DC (%)^∗^	EE (%)^∗^	PS (nm)^∗^	PDI^∗^	ZP (mV)^∗^
FU-NE1	95.36 ± 0.31	94.36 ± 0.51	197.23 ± 2.87	0.278 ± 0.076	+19.1 ± 0.79
FU-NE2	96.59 ± 0.44	93.59 ± 0.44	176.26 ± 1.18	0.166 ± 0.056	−17.2 ± 0.65
FU-NE3	98.26 ± 0.35	91.07 ± 0.61	125.76 ± 1.62	0.137 ± 0.054	−20.9 ± 0.76

^∗^Each value represents mean, *n* = 3 ± SD.

**Table 3:** Density, ST, pH, and viscosity of FU-NEs.

S. no	Formulation	Density (g/cm^3^)	Surface tension (dynes.cm^−1^)	pH	Viscosity (cP)
1	FU-NE1	1.246 ± 0.51	0.4212 ± 0.033	6.96 ± 0.05	2.054 ± 0.65
2	FU-NE2	1.193 ± 0.22	0.4329 ± 0.025	6.92 ± 0.03	1.9242 ± 0.44
3	FU-NE3	1.003 ± 0.06	0.4464 ± 0.014	7.13 ± 0.02	1.1235 ± 0.32

**Table 4:** *In vitro* kinetics of FU release with different FU-NEs (*n* = 3; mean ± SD).

Correlation coefficient (*r*^2^)						
Preparation	Zero order	First order	Higuchi	Hixon Crowell	Korsmeyer-Peppas	Release exponent (*n*)
Pure FU	0.9512 ± 0.13	0.7456 ± 0.27	0.9737 ± 0.43	0.8948 ± 0.81	0.8936 ± 0.80	0.424 ± 0.49
FU-NE1	0.9757 ± 0.16	0.7478 ± 0.72	0.9723 ± 0.12	0.8741 ± 0.41	0.8847 ± 0.36	0.445 ± 0.38
FU-NE2	0.9887 ± 0.12	0.7781 ± 0.67	0.9854 ± 0.34	0.9172 ± 0.32	0.9268 ± 0.18	0.557 ± 0.21
FU-NE3	0.9934 ± 0.43	0.7641 ± 0.36	0.9926 ± 0.61	0.9249 ± 0.13	0.9721 ± 0.52	0.558 ± 0.33

**Table 5:** Stability study of FU-NE3.

Considerations	0 month	1 month	3 months	6 months
DC (%)	98.43 ± 0.32	96.87 ± 0.36	93.99 ± 0.76	89.33 ± 1.95
% EE (%)	91.22 ± 0.46	88.57 ± 0.67	86.90 ± 0.93	83.67 ± 2.76
PS (nm)	125.76 ± 1.62	136.10 ± 2.87	144.12 ± 3.22	161.11 ± 4.92
PDI	0.137 ± 0.054	0.189 ± 0.072	0.208 ± 0.027	0.215 ± 0.086
ZP (mV)	−20.90 ± 0.76	−18.43 ± 0.65	−15.44 ± 1.01	−15.35 ± 1.36
*In vitro* FU released (12 h)	87.23 ± 3.12	88.65 ± 4.90	89.87 ± 5.14	95.33 ± 5.66

^∗^Each value represents mean, (*n* = 3) ± SD.

## Data Availability

The datasets used and/or analyzed during the current study are available from the corresponding authors on reasonable request.
